This article has been retracted.

# Efficiency Measurement of Urban and Rural Logistics Supply Chain System Based on Fuzzy Algorithm

**DOI:** 10.1155/2022/4753343

**Published:** 2022-04-12

**Authors:** Pengliang Qiao

**Affiliations:** ^1^School of Management, Guangzhou College of Technology and Business, Guangzhou 510850, Guangdong, China; ^2^School of Economics and Management, Beibu Gulf University, Qinzhou 535011, Guangxi, China

## Abstract

At this stage, China's logistics industry is developing rapidly and has become one of the important areas of China's economic development. However, there are few techniques for measuring the efficiency of logistics supply chain systems. In order to be able to effectively analyze the efficiency measurement of the urban and rural logistics supply chain system and obtain higher accuracy, using a method derived from analysis of data envelopes, this essay examines the impact elements by establishing a data envelopment analysis model, using compound DEA analysis method and linear regression analysis method. The composite DEA analysis shows that all indicators in the indicator system are positively correlated, and the amount of people working in the field of distribution has the greatest impact on logistics efficiency. The annual average of pure technical efficiency is 0.932, and the annual average of scale efficiency is 0.910. In the eastern region, it is a lower-middle level. The empirical results of changes in the efficiency of the urban and rural logistics industry show that there is a significant positive correlation. This paper also builds a fuzzy algorithm optimization model and designs an overall fuzzy algorithm to solve the LRPPD problem. The simulation results show that the algorithm has good optimization performance, high computational efficiency, and strong convergence speed.

## 1. Introduction

At this stage, China's logistics industry is developing rapidly, and the annual output value in GDP has been increasing, becoming one of the important areas of China's economic development. However, due to the inefficiency of goods in the transportation process, various types of costs continue to increase, and the prices of some commodities even doubled. In order to realize the sustainable development of the logistics market, solving many problems in the logistics supply chain system is the primary task.

The article defines the concepts related to the logistics industry. Based on the data envelopment analysis method, the input and output index system is combined with the experience of the index system selected by the predecessors, and the independent analysis system of the index system is tested by the correlation analysis method. Through the establishment of data envelopment analysis model, a systematic analysis of China's logistics industry was carried out, and the influencing factors were analyzed by using composite DEA analysis method and linear regression analysis method. A fuzzy algorithm model is established and used to analyze the accuracy of this paper.

## 2. Related Work

Judging from the overall development of China's logistics industry, China's logistics industry had a large scale of development and good development prospects at this stage. Many research teams at home and abroad had also conducted in-depth analysis. In [1], the author proposed a path adjustment model in the context of network physical logistics system and minimized the total distribution cost in consideration of road congestion. The static and dynamic models of traffic information transmission network were proposed. In [2], the authors proposed a solution for selecting a logistics provider. The study provides a framework to promote efficiency. In [3], the author studied the traditional logistics model to build an intelligent logistics system based on wireless network technology. Experimental research proved that based on the traditional logistics model, the latest wireless network technology can effectively realize the construction of intelligent logistics system. In [4], the authors studied typical production logistics execution processes and used system dynamics to design cost-effective IoT solutions. The paper used sensitivity analysis to study internal and external production logistics processes and evaluated the best IoT solutions. In [5], the author proposed a hybrid cuckoo search (HCS) algorithm based on optical optimization (OO), particle swarm optimization (PSO), and cuckoo search (CS) to study and optimize the logistics distribution system. The simulation results showed that the algorithm is superior to the traditional algorithm in optimizing the solution, the average solution, the time, and the duration of the search optimal solution.

Fuzzy algorithms can be useful in diverse domains. In [6], scholars applied fuzzy algorithms to video control and proposed an FDASH rate adaptation scheme. In [7], the writer employed the vague algorithm to the medical field and proposed a multivariate multiscale fuzzy entropy (MMFE) algorithm. Based on the characteristics of MMFE, the authors achieved an improvement in the classification accuracy of preterm birth and demonstrated its superiority in synthetic and uterine electromyography (EMG) short-term signals in medical measurements. In [8], scholars proposed a new fuzzy agglomerative computing method. This algorithm can enhance the suppression performance of imagery arrow. In [9], the author used fuzzy time series combined with genetic algorithm (GA) to predict the visit of Taiwan tourists. In [10], the authors found that the aggregation results truly reflect the relationships in the dataset. The experimental results show that entropy theory-based detection of conceptual drift is valid and sensible.

At present, there are few studies on the efficiency of urban and rural logistics supply chain system. This paper proposes a novel research direction based on fuzzy algorithm technology. This technology can effectively improve the efficiency of rural logistics supply chain system and provide a perfect and improved logistics industry. It can also provide new ideas for academic research related to the logistics industry [11–15].

## 3. Method

### 3.1. Urban and Rural Logistics Related Theory

#### 3.1.1. Urban and Rural Logistics Concept

The most important part of rural logistics is agricultural product logistics. Agricultural product logistics refers to the process of transporting agricultural and sideline products produced by farmers as transportation objects, through a series of circulation links such as processing, packaging, and warehousing, from rural areas to urban consumption sites. At present, the urban and rural logistics infrastructure is backward, the information platform construction is not perfect, the circulation cost is high, and the circulation efficiency is low. The introduction of urban logistics is in response to the challenges posed by urbanization and explosive growth of urban transport worldwide. It proposes a series of measures to improve the efficiency of urban goods circulation, thus achieving the city's sustainable development strategy. Urban logistics system refers to the logistics system that serves the city, it serves the needs of urban economic development and refers to the physical flow of goods in the city's internal logistics system. The urban logistics operation system includes all relevant parts of the urban transportation sector and integrates all logistics services.  Figure 1 is a multilevel service supply chain system.

The city and the countryside are a unified whole, and there are close links between the two in terms of economy, society, and culture. Urban and rural logistics mainly have the characteristics of many logistics nodes, short transportation distance, and small transportation batches. The transformation of integration, taking the road of urban and rural coordination and harmonious development, can avoid blind movements, promote the sustainable development of urban and rural economic construction in an orderly and efficient manner, and then conform to the development trend and requirements of modern society.

#### 3.1.2. Urban and Rural Logistics Integration Theory

The main task of urban and rural logistics is to actively promote the construction of a distribution network system for consumer goods and agricultural materials in counties, townships, and villages; integrate and utilize existing logistics resources; further improve infrastructure such as storage, transshipment, docking, and unloading; strengthen service network construction; and improve joint distribution capabilities. The core of urban and rural logistics system development means that the logistics industry focuses on the service functions of urban and rural entities, undertakes the requirements of new urbanization and agricultural modernization for logistics services and quality, and better integrates with the urban and rural industrial chain links. The development provides high-quality and efficient systemized services and ultimately achieves a win-win situation for urban and rural cooperation. The urban-rural logistics integration is proposed in the context of the urban-rural dual structure impeding the harmonious development of urban and rural areas. The purpose is to eliminate the urban and rural “island” phenomenon and to coordinate the urban and rural areas to maximize the overall benefits of the global logistics system.  Figure 2 shows the network structure supply chain structure.

#### 3.1.3. Supply Chain Overview

With the development of economic globalization, competition among enterprises has become increasingly fierce, and supply chains have become a symbol of mutual cooperation between enterprises. Supply chain refers to the network chain structure formed by upstream and downstream enterprises involved in the activities of providing products or services to end users in the production and circulation process. The emergence of the supply chain model has also led to rapid development of enterprises. Since the emergence of the supply chain model, the concept of service has been included, but in the previous supply chain field, more attention was paid to the manufacturing field. The research on service supply chain is still in the initial stage. Service supply chain involves many fields, and there is still no universally accepted definition of service supply chain. The service supply chain at this stage is very different from the beginning of the supply chain. The main body of the basic structure of the supply chain is mainly divided into suppliers, manufacturers, distribution companies, retail companies, and consumers. The initial supply chain is mainly to manufacture products, while the service supply chain participates in the service process of products, and the production and consumption of services occur at the same time. Supply chain is a link in the transportation of products, and the concept of logistics supply chain emerges when products are transported to all parts of the world. There is no doubt that the essence of the logistics supply chain is to provide transportation services. In the construction of service supply chain, the most critical point is that enterprises need to consider not only their current interests, but also their own long-term development. The logistics supply chain takes the customer's logistics needs as the starting point, manages related information, and forms a network model between the initial supplier of the product and the demand from the final customer, which reduces service costs and improves service efficiency.

### 3.2. Logistics Efficiency Measurement Model Based on Data Envelopment Analysis (DEA)

#### 3.2.1. Fixed-Scale Compensation DEA Model—CCR Model

The C2R model is the most basic model of DEA. Give it the appropriate weight *v*, u to build a linear plan; then,

(1) $$\begin{array}{c} X_{i}={\left(X_{1i},X_{2i},\ldots ,X_{mi}\right)}^{T},\\ Y_{i}={\left(Y_{1i},Y_{2i},\ldots ,Y_{ni}\right)}^{T}. \end{array}$$

The efficiency of complex systems is studied and analyzed by weighting each input and output variable. Let *u* be the weight of *X*_*i*_ and *v* the weight of *Y*_*i*_; then,

(2) $$\begin{array}{c} U={\left(u_{1},u_{2},\ldots ,u_{m}\right)}^{T},\\ V={\left(v_{1},v_{2},\ldots ,v_{n}\right)}^{T}. \end{array}$$

The basic efficiency formula is

(3) $$\begin{array}{c} h_{j}=\frac{\sum_{n=1}^{n}U_{n}Y_{nj}}{\sum_{m=1}^{m}V_{m}X_{mj}},\;j=1,2,\ldots ,s, \end{array}$$

where *U* makes *h*_*j*_ ≤ 1(*j*=1,2,…, *s*) by selecting the appropriate weight coefficient *V*. If the weight coefficient is used as a variable,

(4) $$\begin{array}{c} \max h_{0}=\frac{u^{T}Y_{0}}{v^{T}X_{0}}\\ \text{s}.\text{t}\left\{\begin{array}{c} \frac{u^{T}Y_{0}}{v^{T}X_{0}}\leq 1\\ u\geq 0,v\geq 0. \end{array}\right. \end{array}$$

Add the remaining variables *S*^+^, *S*^−^, and perform a dual transformation, where *θ* is a scalar, indicating the efficiency of the DMU. When *θ* = 1, *S*^+^ = *S*^−^ = 0, the decision unit is valid for DEA. At this time, the technology and the scale are effective.

#### 3.2.2. Variable Scale Compensation DEA-BCC Model

The BC2 model adds new constraints to the original C2R model:

(5) $$\begin{array}{c} \sum_{i=1}^{n}\lambda_{i}=1. \end{array}$$

The solution method, such as the C2R model, gives the optimal solution *θ*. When *θ* = 1, *S*^+^ = *S*^−^ = 0, the decision unit is valid for DEA. At this time, the technical efficiency is 1, and the decision unit has reached the best combination of input and output. When *θ* = 1, *S*^+^ ≠ 0, *S*^−^ ≠ 0, the decision unit is valid for weak DEA, and the technical efficiency of the decision unit is not optimal at this time.

### 3.3. Fuzzy Clustering Algorithm Model

Fuzzy algorithms are intelligent algorithms. When we do not have a deep understanding of the model of the system, or when objective reasons prevent us from conducting in-depth research on the control model of the system, intelligent algorithms often play a small role. At this time, we need to use fuzzy algorithms. Common fuzzy algorithms include mean blur, Gaussian blur, and so on. We obtain *n* samples of unknown categories *X*_1_, *X*_2_, *X*_3_,…, *X*_*n*_ from a sample space S; then, the clustering process can be expressed as follows: for each sample *X_i_* (*i*=1, 2,..., *n*), how to make it fall into one of the m regions of S, and *X_i_* only falls into one of the regions is the first problem to be solved. The division of the sample satisfies

(6) $$\begin{array}{c} \left\{\begin{array}{c} S_{1}\cup S_{2}\cup S_{3}\cdots \cup S_{m}=S,\\ S_{i}\cap S_{j}=\emptyset ,\;\forall i\neq j. \end{array}\right. \end{array}$$

#### 3.3.1. Similarity Measurement

(7) $$\begin{array}{c} d\left(X_{i},X_{j}\right)=\sqrt{{\left(x_{i1}-x_{j1}\right)}^{2}+{\left(x_{i2}-x_{j2}\right)}^{2}+\cdots +{\left(x_{il}-x_{jl}\right)}^{2}}\\ d_{M}\left(x_{i},x_{j}\right)=\sqrt{{\left(x_{i}-x_{j}\right)}^{T}\Sigma^{-1}\left(x_{i}-x_{j}\right)}\\ S\left(X_{i},X_{j}\right)=\frac{X_{i}^{T}X_{j}}{\left\|X_{i}\right\|\cdot \left\|X_{j}\right\|},d_{T}\left(X_{i},X_{j}\right)=\frac{X_{i}^{T}X_{j}}{X_{i}^{T}X_{i}+X_{j}^{T}X_{j}-X_{i}^{T}X_{j}}, \end{array}$$

where *d* is the Euclidean distance. Euclidean distance is the simplest and most commonly used side. If the multidimensional space has the same scale concept in all directions, the above formula can be used directly as the similarity measure. Otherwise, the weighted Euclidean distance can be used and expressed as $d\left(X_{i},X_{j}\right)=\sqrt{\sum_{k=1}^{l}\alpha_{k}{\left(x_{ik}-x_{jk}\right)}^{2}}$, where *α*_*k*_ is a weighting coefficient. *d*_*M*_ is the Mahalanobis distance square of the samples *X*_*i*_ to *X*_*j*_, where ∑^−1^ is the inverse of the covariance matrix of each sample vector in the corresponding sample category.

## 4. Experiment

### 4.1. Data Source

In this paper, data from the eastern region including “Beijing, Tianjin, and Hebei” and “Yangtze River Delta” were selected. Therefore, the data covered in this paper are also published data for these regions.

This paper uses statistics on the personnel working in the freight, storage, and mailing sectors at the end of the year in each province as an indicator of the amount of personnel working in the freight forwarding sector. These include the number of employees engaged in road transport, water transport, shipping, pipeline transport, handling and other transport services, warehousing, and postal services. This paper selects the total social fixed assets investment of transportation, warehousing, and postal industries in various provinces and cities as the index data of “logistics fixed assets investment.” Since the fixed-asset investment amount of the whole society. The fixed asset investment price indices in the provinces and municipalities' respective statistical almanacs are expressed in current year prices. In this paper, we use 2011 for the reference period and the fixed asset investment price indices of the relevant years in each province and municipality in order to avoid price differences between years.

### 4.2. Evaluation System

According to the relevant theories and contents of urban and rural logistics integration, combined with the principle of evaluation index construction, the urban and rural logistics integration evaluation index system is finally obtained, including four first-level indicators and twelve second-level indicators, as shown in Table 1.

Tables 2 and 3 are the weight of logistics operation and the weight of logistics platform, respectively. The higher the weight, the greater the importance.

### 4.3. Evaluation Method

#### 4.3.1. Indicator Test

Factor profiling is used to lower the level of the dimensions of most variables, condensing the majority of variables into several common factors and finally using common factors instead of all variables to explain, which requires a certain correlation between the variables; otherwise, the variables are mutually independent. It is impossible to extract common factors for factor analysis. When operating with SPSS software, the KMO test and the Bartlett sphericity test are generally used to test the correlation.

#### 4.3.2. Dimensionless Processing of Raw Data

Since there is no comparability between the indicators, standardization is required to eliminate the influence of the indicator dimension. The basic principle is new data = (raw data − mean)/standard deviation. Suppose there are *n* evaluation objects and *m* quantitative evaluation indicators, and the raw data of the *i*-th object with respect to the *j*th index is *a*_1_. The standardization process is *b*_1_, where *A*_*j*_ and *B*_*j*_ represent mean and criterion error of the *j*-th indicator for those evaluated.

## 5. Results

### 5.1. Analysis of the Overall Change of TFP and Its Decomposition Efficiency in Logistics Industry

This section adopts the output-oriented DEA-Malmquist production efficiency measurement model and the data processed in the previous article and uses relevant analysis software to calculate. The dynamic change value of logistics industry efficiency in China from 2011 to 2018 is shown in Figure 3.

#### 5.1.1. Analysis of the Total Factor Productivity Index

In 2011–2018, China's logistics industry TFP index increased by an average of 3.3%, and the overall growth was relatively uniform. The growth of TFP generally represents the growth of output growth due to technical or management reasons when certain productive inputs are unchanged. Therefore, China's logistics industry includes logistics enterprises and national logistics management departments for logistics industry operation management technologies and new technologies. The increasing application degree has greatly promoted the development of China's logistics industry. However, in the past 8 years, the logistics industry's skilled level of efficiency fell by 3.1% on average. The performance of pure technology has decreased by 2.9%, the scale efficiency has decreased by 0.2%, and the technological progress index has increased by an average of 6.6%. It is possible to introduce technological progress to a certain extent. A certain coverage, on the one hand, reflects that China's logistics industry is more avant-garde in the development and application of new technologies or new models, but in the application phase of new technologies, it does not pay attention to benefits, and the large investment in application research and development is exchanged for inefficient small gains; on the other hand, it reflects that technological progress can significantly increase total factor productivity.

#### 5.1.2. Analysis of Pure Technical Efficiency and Scale Efficiency

From 2011 to 2018, the pure and simple gross technical economy of China's distribution chain declined by an average of 2.9%. From the line graph, the true value of net technological efficiency is below 1 in all years except 2012, 2014, and 2018, that is, without considering economies of scale. In this case, the pure technical efficiency of China's logistics industry was ineffective in these five years, reflecting the inefficient management methods of logistics enterprises and logistics industry management departments in these five stages, and the management methods and technological progress are not synchronized.

### 5.2. Measurement and Analysis of Urban and Rural Logistics Industry

#### 5.2.1. Horizontal Measure

A detailed analysis of the overall technical efficiency of the material flow industry provides a clear picture of the trends in the region's material flow industry. The following section continues to compare the combined technical efficiency of the logistics industry, yielding the following graphical view. It can be seen from Figure 4 that the logistics industry of the “Yangtze River Delta” has developed steadily and has a tendency to rise slowly in the past 8 years. The “Beijing-Tianjin-Hebei” has fluctuated greatly and has shown a downward trend since 2014. Compared with the two major economic zones, there are still significant gaps in the overall development of the logistics industry.

It can be seen from Figure 5 that the overall development trend in the eastern region is relatively stable, with large fluctuations in Beijing, Tianjin, and Hebei provinces. Among them, Beijing is higher than the eastern region in 2016 and 2017 and lower than the eastern region in other years; Tianjin's comprehensive technical efficiency before 2013 is effective, but it has continued to decline since 2014; even in 2018, it was only 0.508; the comprehensive technical efficiency of Hebei Province in the past 8 years was relatively stable, similar to the overall development trend in the eastern region.

#### 5.2.2. Longitudinal Measure

Comparing the average value of the Beijing-Tianjin-Hebei region and the eastern region, the average annual growth rate of Beijing is 4.5%, the average annual growth rate of Hebei Province is 5%, and the average annual growth rate of Tianjin is negative. The overall average annual growth rate is 0.9%. It can be seen from Figure 6 that the eastern region has been on an upward trend since 2015 to 2016 and has experienced varying degrees of decline.

From comparative findings, the development trends of the two regions from 2001 to 2018 are basically similar, but the average annual growth rate is slightly lower in the triangle region. Based on the analysis above, causes of low productivity are not only purely technically inefficient, but also low in scale efficiency. Therefore, even if the Beijing-Tianjin-Hebei region has a relatively complete material base such as logistics facilities, it is difficult to sustain growth and even cannot maintain growth.

### 5.3. Empirical Analysis of Influencing Factors of Urban and Rural Logistics Efficiency Changes

Based on the regression model, this paper uses Eiews6.0 measurement software to analyze the regression model corresponding to total and solely based upon our technical expertise. The obtained empirical results are shown in Tables 4 and 5.

1. Economic development level coefficients of LGDP are all positive, and both are significant at the level of 1% (0.01). This shows that the efficiency of urban and rural logistics industry has a significant positive correlation with the level of economic development. For every 1 percentage point increase in economic development level, the total technical efficiency of the urban and rural logistics industry will be increased by 0.127464 percentage points, and the pure technical efficiency of 0.024423 percentage points.
2. For logistics resource utilization, the three coefficients of LU are negative, and both are significant at the level of 1% (0.01). An increase in the rate of urban and rural material flows utilization does not improve the productivity of the material flows sector. On the contrary, for every 1% rise in the rate of resource use in urban and rural areas, the total technical inefficiency of the urban and rural logistics industry will be significantly reduced by 0.225264 percentage points and the peak pure social economy by 0.048304 percentage points.

### 5.4. Fuzzy Algorithm Model Optimization Solution Analysis

The following parameters are used: the maximum number of iterations is max_iter = 500, the tabu length *L* = 5, the number of candidate solutions = 60, and the penalty value of the infeasible line is *M* = 3000. The algorithm is implemented by Matlab7.1, and it is solved 10 times in CPU1.8 G and memory 512 M. The calculation results are shown in Table 6.

It can be seen from Table 6 and Figure 7 that the high-quality solution is obtained in the 10 solutions of the example using the fuzzy algorithm. For the positioning of integrated distribution and collection, the average mileage of the transportation route is 552.6 (km), and the average number of vehicles used is 7.8. Among them, the solution obtained in the sixth solution has the highest quality, and its total mileage is 528 (km). The calculation result of the fuzzy algorithm is also stable. In the 10 times of solving, the total mileage of the worst solution is only 9.2% higher than the best solution. From the perspective of computational efficiency, the average calculation time of 10 solutions is only 18.5 s, and the calculation efficiency is also high. It can be seen from the figure that the fuzzy algorithm for solving the integrated distribution and collection of urban and rural logistics has the following characteristics:

The quality of the solution is continuously improved with the progress of the search process. In the initial stage, the quality of the solution is improved rapidly; as the search process continues, the quality of the solution is gradually slowed down until it reaches the optimal level. The quality of the solution is no longer improved. The good optimization performance of the algorithm is fully shown from the figure, which guarantees a good calculation result and also has a high convergence speed.

## 6. Conclusions

In order to be able to effectively analyze the efficiency measurement of the urban and rural logistics supply chain system and obtain higher accuracy, based on the data envelopment analysis method, this paper uses the compound DEA analysis method and the linear regression analysis method to analyze the influencing factors.

In the 8 years of China's logistics industry, TFP increased by 3.3%, and the growth was relatively flat. The growth rate of the technology progress index reached 6.6%, which masked the decline of technical efficiency, indicating that the key technology research and development of China's logistics industry has achieved certain results. According to the composite DEA analysis, all the indicators in the indicator system show a positive correlation. The number of employees in the logistics industry has the greatest impact on logistics efficiency, but the application of different provinces is also different.

The average annual technical efficiency of the regional logistics industry is 0.849, the annual average of pure technical efficiency is 0.932, and the annual average efficiency of scale is 0.910, which is a moderately lower level in the eastern region. Overall, the region still has development potential. From a vertical perspective, the logistics industry in the Beijing-Tianjin-Hebei region is developing at a slow pace. The annual average of the factor-factor productivity change index is 1.009, and the efficiency growth rate is only 0.9%, far below the average level in the eastern region.

Combining the empirical results of urban and rural logistics industry efficiency changes and regional differences, we can draw the following conclusions: there was a positive and substantial association with the economic development level and location advantage and logistics industry efficiency. There is a certain negative correlation between logistics resource utilization rate, logistics talents and industrial structure, and logistics industry efficiency. According to the degree of division, the location advantage has the greatest improvement in the efficiency of the logistics industry, followed by the level of economic development, both of which are the contributing factors to the efficiency changes of the urban and rural logistics industry.

The fuzzy algorithm optimization model is constructed, and the fuzzy algorithm for solving the LRPPD problem is designed as a whole. The simulation results show that the algorithm has good optimization performance, high computational efficiency, and strong convergence speed. The example shows that the algorithm has local optimization and overall optimization performance, greatly improves the quality of optimization, and has the advantage that traditional methods cannot match for solving medium- and large-scale problems.

## Figures and Tables

**Figure 1:** Multilevel logistics service supply chain.

**Figure 2:** Basic network structure.

**Figure 3:** National annual total factor productivity and its decomposition efficiency index change line chart.

**Figure 4:** Comparison of comprehensive technical efficiency of logistics industry in Beijing, Tianjin, and Hebei provinces and eastern regions in 2011–2018.

**Figure 5:** Comparison of comprehensive technical efficiency of “Beijing-Tianjin-Hebei” and “Yangtze River Delta” logistics industry in 2011–2018.

**Figure 6:** Comparison of TFP values between Beijing-Tianjin-Hebei and Yangtze River Delta.

**Figure 7:** Total mileage and calculation times of integrated distribution and collection routes.

**Table 1:** Urban and rural logistics integration evaluation index system.

Aims	Primary indicator	Secondary indicators
Urban and rural logistics integration development level index system	Urban and rural economic development level (X1)	Logistics industry added value (X11)
		Total investment in fixed assets (X12)
		Gross regional product (X13)
	Logistics infrastructure construction level (X2)	Cargo transportation volume (X21)
		Highway mileage (X22)
		Railway mileage (X23)
	Urban and rural information development level (X3)	Total post and telecommunications business (X31)
		Internet access (X32)
		Mobile phone year-end users (X33)
	Urban and rural logistics organization scale (X4)	Number of employees related to logistics (X41)
		Number of logistics companies (X42)
		Number of supply and marketing cooperatives (X43)

**Table 2:** Weights of logistics operations.

Operating systems	Logistics main body	Channels	Functions
Logistics main body	1.03	3.34	4.98
Channels	0.31	1.02	1.54
Functions	0.23	0.69	1.06

**Table 3:** Weights of logistics platforms.

Platform	Facilities	Policies	Technology	Talent
Facilities	1.01	0.68	2.2	3.1
Policies	1.53	1.02	2.23	2.8
Technology	0.42	0.47	1.06	2.3
Talent	0.31	0.37	0.45	1.04

**Table 4:** Total technical efficiency model regression results.

Interpret variable	Coefficient estimate	Standard error	Z statistic	*P* value
C	1.661816	0.549122	3.026318	0.0025
LGDP: The level of economic development	0.127464	0.022242	5.730889	0.0001
LU: Logistics resource utilization	−0.225264	0.046595	−4.834524	0.0001
LQ: Location advantage	0.180111	0.101763	1.769900	0.0767
LP: Logistics person	0.002664	0.002319	1.148531	0.2507
IS: Industrial structure	−1.934998	1.129634	−1.712942	0.0867

**Table 5:** Pure technical efficiency model regression results.

Interpret variable	Coefficient estimate	Standard error	Z statistic	*P* value
C	1.330886	0.138834	9.586198	0.0001
LGDP: The level of economic development	0.024423	0.005623	4.343247	0.0001
LU: Logistics resource utilization	−0.048304	0.011781	−4.100319	0.0001
LQ: Location advantage	0.022034	0.025729	0.856384	0.0918
LP: Logistics person	−0.000207	0.000586	−0.352349	0.7246
IS: Industrial structure	−0.740099	0.285604	−2.591350	0.0096

**Table 6:** Fuzzy algorithm calculation results.

Calculation order	Total mileage	Number of vehicles	Number of iterations	Calculation time
1	545	8	252	18
2	576	9	330	20
3	558	8	374	20
4	567	8	310	20
5	539	7	238	17
6	529	7	292	18
7	549	8	394	20
8	567	8	206	17
9	558	8	228	17
10	539	7	246	18
Average	552.6	7.8	287	18.5

## Data Availability

This article does not cover data research. No data were used to support this study.

## References

[1] Lai M., Yang H., Yang S., Zhao J., Xu Y. (2017). Cyber-physical logistics system-based vehicle routing optimization. *Journal of Industrial and Management Optimization*.

[2] Yazdani M., Zarate P., Coulibaly A., Zavadskas E. K. (2017). A group decision making support system in logistics and supply chain management. *Expert Systems with Applications An International Journal*.

[3] Ouyang Q., Zheng J., Wang S. (2019). Investigation of the construction of intelligent logistics system from traditional logistics model based on wireless network technology. *EURASIP Journal on Wireless Communications and Networking*.

[4] Qu T., Thürer M., Wang J. (2017). System dynamics analysis for an internet-of-things-enabled production logistics system. *International Journal of Production Research*.

[5] Chen X., Wang J. (2016). A novel hybrid cuckoo search algorithm for optimizing vehicle routing problem in logistics distribution system. *Journal of Computational and Theoretical Nanoscience*.

[6] Vergados D. J., Michalas A., Sgora A., Vergados D. D., Chatzimisios P. (2016). Fdash: a fuzzy-based mpeg/dash adaptation algorithm. *IEEE Systems Journal*.

[7] Ahmed M., Chanwimalueang T., Thayyil S., Mandic D. (2016). A multivariate multiscale fuzzy entropy algorithm with application to uterine EMG complexity analysis. *Entropy*.

[8] Zhang X., Sun Y., Gang W., Qiang G., Zhang C., Chen B. (2016). Improved fuzzy clustering algorithm with non-local information for image segmentation. *Multimedia Tools and Applications*.

[9] Sakhuja S., Jain V., Kumar S., Chandra C., Ghildayal S. K. (2016). Genetic algorithm based fuzzy time series tourism demand forecast model. *Industrial Management & Data Systems*.

[10] Zhang B., Shan Q., Wei W., Dan W., Lei X. (2016). Data stream clustering based on fuzzy C-mean algorithm and entropy theory. *Signal Processing*.

[11] Li Q., Wu G. (2021). ERP system in the logistics information management system of supply chain enterprises. *Mobile Information Systems*.

[12] Abd el-gawad A. F., Zaki S., Kamal E. (2021). A survey on machine learning techniques for supply chain management. *American Journal of Business and Operations Research*.

[13] Pustokhina I. V. (2020). Blockchain technology in the international supply chains. *International Journal of Wireless and Ad Hoc Communication*.

[14] Pan C., Liu M. (2021). Optimization of intelligent logistics supply chain management system based on wireless sensor network and RFID technology. *Journal of Sensors*.

[15] Sudan T., Taggar R. (2021). Recovering supply chain disruptions in post-COVID-19 pandemic through transport intelligence and logistics systems: India’s experiences and policy options. *Front. Future Transp.*.

